# Cutaneous mast cell tumor (Mastocytoma): Cyto*-* histopathological and haematological investigations

**DOI:** 10.1186/1746-1596-9-9

**Published:** 2014-01-20

**Authors:** Ehsan Hosseini, Behnam Pedram, Ali Mohammad Bahrami, Mohammad Hossein Jaberi Moghaddam, Javad Javanbakht, Fatemeh Emami Ghomi, Najme Jaberi Moghaddam, Mobin Koohestani, Radmehr Shafiee

**Affiliations:** 1 Faculty of Para Veterinary Medicine, Ilam University, Ilam, Iran; 2 Department of Pathobiology, Susangerd Branch, Islamic Azad University, Susangerd, Iran; 3 Graduate, Faculty of Veterinary Medicine, Urmia University, Urmia, Iran; 4 Department of Pathobiology, Faculty of Veterinary Medicine, Tehran University, Tehran, Iran; 5 Graduate, Faculty of Medicine, Iran University of Medical Sciences, Tehran, Iran; 6 MSc, Clinical Biochemistry, Tarbiat Modares University, Tehran, Iran; 7 Graduate, Faculty of Veterinary Medicine, Tehran University, Tehran, Iran

**Keywords:** Cytology, Pathology, Dog, Mast cell tumor, Grading

## Abstract

Cutaneous mast cell tumours (MCTs) are the most common skin tumours in dogs. Due to the prevalence of canine MCTs and the variable biologic behavior of this disease, accurate prognostication and a thorough understanding of MCT biology are critical for the treatment of this disease. A cytologic diagnosis of mast cell tumor with evidence of prior hemorrhage was made, and the masses were surgically removed. Cytological evaluation of fine-needle aspirates from the cutaneous mass from the axillary comprised many well-differentiated, highly granulated mast cells with moderate numbers of eosinophils. Nuclei were varied in size and shape with high nuclear’to’cytoplasmic ratio, prominent nucleoli, marked atypical and mitotic figures. Microscopically, mass consisted of sheets of neoplastic round cells that formed nonencapsulated nodules in the dermis and infiltrated into the adjacent dermal collagen, and also there was diffuse subcutis invasion of round to pleomorphic tumor cells. Tumor cells had moderate to abundant cytoplasm, round to ovoid nuclei with scattered chromatin, and mitotic figures. In this tumor, cytoplasmic granules showed atypical metachromasia. In addition, eosinophils were scattered among the mast cells at the periphery of the nodules. The presence of eosinophils and the observation, at high magnification, of cells with cytoplasmic metachromatic granules. Invasion of the deep subcutaneous fat or cutaneous muscles were a common feature of grade III tumour. Finally, a diagnosis of grade III cutaneous mast cell tumor was made.

**Virtual slides:**

The virtual slide(s) of this article can be found here: http://www.diagnosticpathology.diagnomx.eu/vs/4755249151157024.

## Background

Mast cell tumors (MCTs) are highly invasive and metastatic and are the most frequent round cell tumors in dogs, comprising 16–21% of all cutaneous tumors diagnosed [1,2], and are the most common skin tumors in dogs [3], representing about 7% to 21% of all dog skin tumors and 11% to 27% of malignant skin tumors in this species [4]. Canine MCTs have variable biologic behaviors, ranging from solitary benign masses that can be cured with surgery alone to systemic and potentially fatal metastatic disease [5], and are always considered potentially malignant, but their true metastatic potential is not entirely known [6].

Round cell tumors consist of discrete cells that are round to oval rather than fusiform. Included in this group are mast cell tumor, histiocytoma, lymphosarcoma (including reticulum cell sarcoma) and transmissible venereal tumor. The differential diagnosis of round cell tumors by histologic examination without concomitant cytologic characterization may, in some instances, depend more on age of animal, growth rate, location of tumor, number of tumors and lymph node involvement rather than histologic criteria. Mastocytosis is a rare group of diseases characterized by abnormal proliferation and infiltration of mast cells within the tissues. The skin is most frequently involved but mast cells also accumulate in the bone marrow, gastrointestinal tract, lymph nodes, spleen, and liver. Mast cell tumors in association with oncocytes thus should be considered supportive evidence of an FNA diagnosis of adenolymphoma. Mastocytosis should be considered in the differential diagnosis of urticaria and solitary mastocytomas may remain active into adolescence, raising concern for systemic progression [7-13].

MCTs are most often graded histologically by the scheme described by Patnaik et al. [14]. Tumours of grade I are circumscribed, mainly dermal in location, and consist of well-differentiated mast cells with prominent metachromatic cytoplasmic granules. Poor cellular differentiation, aggressive growth pattern, moderate to high mitotic activity, mitotic atypia and sparse to absent cytoplasmic granulation are the major features of grade III tumours. Grade II MCTs constitute an intermediary form between the two other grades, but they tend to infiltrate more deeply than grade I neoplasms [14,15]. MCTs are routinely diagnosed by cytology and histopathology.

## Case presentation

### Animal ethics

The animal was placed in shade, in standard conditions, water ad libitum, and without restriction of movement according to the guidelines of Institutional Animal Ethical Committee of the Tehran University of Animal Science, Iran. Surgery was performed under aseptic conditions and sedation by injection of Xylazine hydrochloride (0.05 mg/kg) followed by 2% Lignocaine hydrochloride.

### Clinical case reports

In October 2013, a 5-year-old, 7 kg, female black terrier dog was presented to the clinic at the college of Veterinary Medicine, university of Tehran, with a growing mass around axillary and mobility problems related to the mass, and euthanasia was applied upon the owner’s request and also taking into consideration the age of the animal and the size of the mass. The mass spreading into subcutis is of proximal right front leg, was of 2.8 × 2.5 cm size and 185 g weight (Figure 1). The mass was surgically resected and an impression smear of the tissue was prepared and stained with Giemsa. The rest of the tissue was subjected to histopathologic evaluation.

**Figure 1:** **Cytohistophatology of dermal mass from the axillary of the dog.** Representative photomicrographs of mass cell tumuor of Patnaik grade. **(A and B)** grade III. High-grade mast cell tumour was characterized by highly pleomorphic tumour cells with a high mitotic index, anisokaryosis and infiltration of the surrounding dermis and subcutis. Haematoxylin and eosin stain. Bar, 50 μm. the smears show n were prepared at the initial presentation and stained with Wrigth-Giemsa solution. Histopathologically, The presence of eosinophils and the observation, at high magnification, of cells with cytoplasmic metachromatic granules and also, neoplastic cells often exhibited an aggressive behavior, high cellularity, cellular pleomorphism, and various morphologic patterns. Eosinophils are present at the periphery of the mass (Figure 1**C** and **D**, H&E, 400x).

One formalin-fixed, paraffin wax-embedded section of each neoplasm was stained with haematoxylin and eosin (HE). Tumour was classified independently by two pathologists in order to confirm the diagnosis according to the WHO criteria [16]. Also tumour was graded according to the criteria proposed by Patnaik et al. [14] and Kiupel et al. [17], as well, moderately or poorly differentiated (grades I, II or III, respectively) [14,17]. These criteria included the following histomorphological features: extent of tumour (invasiveness), cellular morphology, size of cytoplasmic granules, mitotic activity and stromal reaction. Invasiveness was assessed as follows: non-invasive (tumours confined to the superficial dermis and interfollicular spaces); moderately invasive (tumours with lower dermal and limited subcutaneous tissue invasion); highly invasive (tumours with massive infiltration of subcutaneous and deep tissue). Mitotic activity was assessed on toluidine blue-stained sections, five high power fields (hpfs) being evaluated in each case with a × 40 objective. The data were expressed as mean number of mitoses per hpf (mitotic index) and tumours were classified according to the following grading system: 0 (mitotic figures absent); 1 (mitotic index ranging from 0 to 2 mitoses/hpf); 2 (mitotic index > 2/hpf). Invasiveness and mitotic activity assessment were used to define the histological grade, and also as individually evaluated parameters.

### Hematological findings

A complete blood work was performed. No changes were noticed in the erythrogram, however, leukogram changes included leukocytosis (55,245 leukocytes/μL), neutrophilia (27,644 neutrophils/μL) with mild regenerative left shift (4,376 band cells/μL).

### Cytological findings

Cytological examination indicated mast cells with numerous metachromatic stained granules. Nuclei were varied in size and shape with high nuclear’to’cytoplasmic ratio, prominent nucleoli, marked atypical and mitotic figures. The background was filled with granules from ruptured cells and a moderate eosinophils were also present (Figure 2A and 2B).

**Figure 2:** **Macroscopical examination of a cutaneous cell tumor in a black terrier.** The mass spreading into subcutis is of proximal right front leg.

### Histopathological findings

Histopathologically, MCT tumour cells were less well circumscribed by connective tissue and neoplastic cells often exhibited an aggressive behavior, high cellularity, cellular pleomorphism, and various morphologic patterns.

However, in some regions of the tumor tissue shows neoplastic cells extending into the subcutis. Neoplastic cells had distinct cell borders and widely variable amounts of pale to brightly eosinophilic cytoplasm. Furthermore, tumour had neoplastic cells containing numerous fine eosinophilic to basophilic cytoplasmic granules consistent with mast cell granules and also highly pleomorphic tumour cells with a high mitotic index, anisokaryosis and infiltration of the surrounding dermis and subcutis were observed (Figure 2C and 2D).

### Pathology *grading* of cutaneous mast cell tumor

In this case is characterized by one or more of the following criteria: at least 3 mitotic figures in 5 hpf, at least 2 multinucleated (2 or more nuclei) cells in 5 hpf, at least 2 bizarre nuclei (highly atypical with marked indentations, segmentation, and irregular shape) in 5 hpf; karyomegaly (ie, nuclear diameters of at least 10% of neoplastic mast cells vary by at least 2-fold). The selected field was it that was most highly mitotically active or had the highest degree of anisokaryosis.

Canine cutaneous MCTs were graded according to the Patnaik and the Kiupel systems [14,17]. Grade III MCT was poorly demarcated accumulations of poorly differentiated mast cells with severe nuclear pleomorphism. Invasion of the deep subcutaneous fat or cutaneous muscles were a common feature of grade III tumour. Finally, a diagnosis of grade III cutaneous mast cell tumor was made.

## Discussion

Dogs are at risk for cutaneous MCT, which accounts for up to 21% of all skin tumours [3]. The diagnosis of MCT by cytology or histopathology is straight forward in the majority of cases, but forming an accurate prognosis is more challenging [5]. Prognostic factors of significance included grading (cytology and histopathology), staging (regional and distant metastases), breed, tumour localisation and treatment (surgery, radiation and chemotherapy). Cytological examination after fine needle aspiration is useful in establishing the diagnosis but histopathology is needed for grading [18]. Cytology often is helpful in the diagnosis of MCTs because of the characteristic appearance of mast cells with routine staining. As is the case with findings from other species, Wright–Giemsa stain resulted in more intensely stained granules in the neoplastic mast cells. The mechanism of the differences in staining is unclear. Several subtypes of mast cells have been identified in humans and dog based primarily on granule contents and biological function.

This study clearly showed a cellular infiltrate of mast cells, mononuclear cells and eosinophils in the thickened, hyperplastic, and hyperkeratinized epidermis. Mast cells and eosinophils, as opposed to the mononuclear cells of delayed hypersensitivity, predominated, suggesting an immediate hypersensitivity reaction. Once activated, mast cells at the edge of a wound are known to release inflammatory mediators within injured tissue by degranulation [19]. Thus, it would seem that immediate hypersensitivity reactions may be responsible for the development of skin lesions due to tumor in dogs. However, the present results suggest that the intense proliferation of mast cells following tumor occurs predominantly in the skin.

The results of this study suggest that cellular proliferation plays a significant role in the progression of canine MCTs. Although the results of this study confirm the results of previous studies that have shown the prognostic significance of cellular proliferation in canine MCTs [14,15,18,19] cellular proliferation should not be evaluated as a single prognostic factor for canine MCTs but should be evaluated in tandem with additional prognostic indicators. Furthermore, the histologic characteristics of the MCT cells in this affected dog was moderate to abundant cytoplasm, round nuclei with scattered chromatin, fibrous stroma, and eosinophil infiltration. Little necrosis was seen.

Several grading systems have been proposed to classify canine mast cell tumors. The system most commonly used classifies the tumor from grades I to III, depending on how well the mast cells are differentiated, mitotic activity, location within the skin, invasiveness, and the presence of inflammation or necrosis, with grade III being the most aggressive (characterized by the presence of undifferentiated, immature mast cells with a high potential for metastasis) [20,21]. In the current case, the presence of multiple large nodules, the extension into the dermis, and the poorly differentiated mast cells could be comparable to grade III described for dogs. Recently, a new 2-tier histologic classification for canine cutaneous tumors has been proposed [22]. This grading system is based on the presence of mitotic figures, multinucleated cells, bizarre nuclei, and karyomegaly to predict biological behavior, likely time to metastasis, new tumor development, and survival time. In the present case, although the neoplasia did not show any of these histological parameters, the presence of multiple cutaneous tumors suggests a malignant behavior. Grade III tumours have a very poor prognosis even with treatment, which might discourage owners from extensive surgery. This may explain the discrepancy in surgery performed in MCT cases of different grades. This result agrees with the findings by Murphy et al. [23] that showed dogs with poorly differentiated tumours had a significantly shorter survival time. These results suggest that all multiple cutaneous MCTs should be treated as individual neoplasms and prognosis should be dependent on individual variables such as grade and not related to the number of tumours present, which was shown not to affect survival. Mitotic index and size were not found to be independent predictors of survival.

## Conclusions

In conclusion, this study described cytohistopathology features of canine cutaneous MCTs of the skin region. The histological features of these tumours would suggest that most should be classified as high-grade MCTs. A cutaneous MCT may be diagnosed on the basis of observing the histopathological pattern described in present study. Moreover, the use of grading system for a tumor type may be helpful in distinguishing this type of neoplasm from other malignancies with similar morphology. Furthermore, this study demonstrated that in canine cutaneous MCTs, may be used as a sensitive prognostic indicator of post-surgical tumour behaviour; in addition, it is related to other histopathological variables that are widely accepted as having prognostic value.

## Competing interests

The authors declare that they have no competing interests.

## Authors’ contributions

EH, BP and AMB participated in the histopathological evaluation, performed the literature review, acquired photomicrographs and drafted the manuscript and gave the final histopathological diagnosis. MHJM, FEGH, JJ, NJM, MK and RSH designed and carried out all the experiments and the principal investigators of the laboratory in which the research were performed and contributed to the interpretation of the data and writing of the manuscript. All authors read and approved the final manuscript.
